The article "Correlation Analysis Between Required Surgical Indexes and Complications in Patients With Coronary Heart Disease" was retracted in 2023. Reasons: compromised peer review; false authorship; unreliable results or conclusions; concerns about the data.

# Correlation Analysis Between Required Surgical Indexes and Complications in Patients With Coronary Heart Disease

**DOI:** 10.3389/fsurg.2022.948666

**Published:** 2022-07-06

**Authors:** Meiyi Tao, Xiaoling Yao, Shengli Sun, Yuelan Qin, Dandan Li, Juan Wu, Yican Xiong, Zhiyu Teng, Yunfei Zeng, Zuoheng Luo

**Affiliations:** ^1^ Department of Nursing, Hunan Provincial People's Hospital (The First-Affiliated Hospital of Hunan Normal University), Changsha, China; ^2^ Department of Respiratory Medicine, Hunan Provincial People's Hospital (The first-Affiliated Hospital of Hunan Normal University), Changsha, China; ^3^ Department of Neurosurgery, Hunan Provincial People's Hospital (The First-Affiliated Hospital of Hunan Normal University), Changsha, China; ^4^ The Third Department of Cardiovascular Medicine, Hunan Provincial People's Hospital (The First-Affiliated Hospital of Hunan Normal University), Changsha, China; ^5^ Clinical Medicine Research Center of Heart Failure of Hunan Province, Changsha, China

**Keywords:** patients with coronary heart disease, preoperative examination, complications of coronary heart disease, vascular lesions, arteriosclerosis, VTE

## Abstract

A total of 215 patients with coronary heart disease (CHD) were analyzed with SPSS. Samples of different genders showed significance in the obtuse marginal branch of the left circumflex branch × 1, the diagonal branch D1 × 1, and the ms PV representation. Patients with left circumflex branch occlusion are more male and tend to be younger. Age displayed a positive correlation with left intima-media thickness (IMT) and right IMT. This indicated that as age increases, the values of left IMT and right IMT increase. Samples of different CHD types showed significance in the obtuse marginal branch of the left circumflex branch × 1, the middle part of RCA × 1, and the middle part of the left anterior descending branch × 1.5. For non-ST-segment elevation angina pectoris with acute total vascular occlusion, the left circumflex artery is the most common, followed by the right coronary artery and anterior descending branch. Ultrasound of carotid IMT in patients with CHD can predict changes in left ventricular function, but no specific correlation between left and right common carotid IMT was found. Samples with or without the medical history of ASCVD showed significance in the branch number of coronary vessel lesions. The value of the branch number of coronary vessel lesions in patients with atherosclerotic cardiovascular disease (ASCVD) was higher than in those without ASCVD. The occurrence of complication is significantly relative with the distance of left circumflex branch × 1, the middle segment of left anterior descending branch × 1.5, and the distance of left anterior descending branch × 1. For patients without complications, the values in the distal left circumflex branch × 1, the middle left anterior descending branch × 1.5, and the distal left anterior descending branch × 1 were higher than those for patients with complications. The VTE scores showed a positive correlation with the proximal part of RCA × 1, the branch number of coronary vessel lesions, the posterior descending branch of left circumflex branch × 1, the distal part of left circumflex branch × 1, and the middle part of left anterior descending branch × 1.5.

The article "Correlation Analysis Between Required Surgical Indexes and Complications in Patients With Coronary Heart Disease" was retracted in 2023. Reasons: compromised peer review; false authorship; unreliable results or conclusions; concerns about the data.

## Introduction

Coronary heart disease (CHD), the most common type and the leading cause of death in cardiovascular disease, is a type of heart disease caused by coronary artery stenosis or occlusion (1). It is common for adults aged 40 years and older and is more common in males. In recent years, this type of disease has been more prevalent at younger age than in the past. The most common symptoms of CHD are chest pain, palpitations, and shortness of breath. SPSS has been widely used in research related to CHD (2, 3). In addition to age, genetic factors, and other uncontrollable factors, high blood pressure, diabetes (4), obesity (5), smoking (6), and other controllable factors are also risk factors for CHD. The study of these influencing factors provides a theoretical and practical basis for the prevention and treatment of CHD (7, 8).

As shown in Figure 1, before surgery, pathological analysis of CHD is used more frequently. Coronary angiography, the most widely used diagnostic method for CHD, may cause physical injury and some complications as well as adverse reactions to patients. What is more, this type of diagnostic method is expensive (9). There are some effective methods for the surgical treatment of CHD, including percutaneous coronary intervention (PCI) and coronary artery bypass grafting (CABG). The disease, however, cannot be cured radically (10, 11). Complications in patients with CHD are caused by damaged systemic blood supply after impaired cardiac function. It includes renal failure, diabetes, heart failure, and other complications (12). Patients with diabetes are more likely to have CHD (13). CHD is the leading cause of death in patients with non-alcoholic fatty liver disease (NAFLD), and the association between them is mediated by a combination of diabetes and body mass index (14). The degree of CAD has relations to an increased risk of stroke, TIA, and systemic embolism (15). Venous thromboembolism (VTE) with CHD is common in a clinic (16), andVTE is easy to occur after CABG (17). Hsa_circ_0001946, hsa-miR-7-5p, and PARP1 as the predictive power of combined biomarkers of CHD and the regulatory axis they constitute may contribute to the prevention of CHD (18). Heart failure has relations with bleeding risk in patients with CHD (19). Preoperative heart failure with preserved ejection fraction was significantly associated with a decrease in 5-year survival after successful CABG (20).

The article "Correlation Analysis Between Required Surgical Indexes and Complications in Patients With Coronary Heart Disease" was retracted in 2023. Reasons: compromised peer review; false authorship; unreliable results or conclusions; concerns about the data.

**Figure 1:** Explanation before and after operation of coronary heart disease.

We analyzed 215 patients who suffered from CHD, with 128 males and 87 females. The study analyzed the obtuse marginal branch of the left circumflex branch, the diagonal branch, and the representative of ms PV (pulmonary valve) by using an independent-sample *t*-test in different ages and sexes. The complications of CHD and family medical history were analyzed by ANOVA and a chi-square test. The study tried to find the correlation between these several variables.

## Methods

### General Description

A total of 215 CHD patients were selected as subjects, with 128 males and 87 females. These patients were admitted to the Department of Cardiology of our hospital from February 2017 to June 2021.

### Inclusion and Exclusion Criteria

Inclusion criteria are as follows:

(1) Age: 32–94 years old;
(2) Voluntarily, one can communicate and agree to data collection.

Exclusion criteria are as follows:

(1) Unconscious; unable to communicate effectively;
(2) Cardiopulmonary dysfunction; the patient's condition is unstable.

## Results

As shown in Table 1, the *t*-test (independent-sample *t*-test) was used to analyze the differences between sexes for the obtuse marginal branch of the left circumflex branch × 1, the diagonal branch D1 × 1, and ms PV. As shown in Table 1, samples of different genders showed significance in the obtuse marginal branch of the left circumflex branch × 1, the diagonal branch D1 × 1, and the ms PV representation. Patients with left circumflex branch occlusion are more male and tend to be younger.

**Table 1:** *t*-Test analysis of sex and obtuse marginal branch of the left circumflex branch × 1, diagonal branch D1 × 1, and ms pulmonary valve representative.

	Gender (mean and standard deviation)		*t*	*p*
	Female (*n* = 87)	Male (*n* = 128)		
82. Obtuse marginal branch of left circumflex branch × 1	1.49 ± 1.06	1.88 ± 1.37	−2.134	0.034*
79. Diagonal branch D1 × 1	1.75 ± 1.29	2.44 ± 1.54	−3.269	≤0.001**
ms pulmonary valve representative	0.99 ± 0.19	0.92 ± 0.22	2.334	0.021*

*p < 0.05; **p < 0.01.

As shown in Table 2, correlation analysis was performed to analyze the correlation between age and intima-media thickness (IMT) of the left common carotid artery and IMT of the right common carotid artery. The Pearson correlation coefficient was used to show the strength of the correlation. From the correlation coefficient and *p*-value in Table 2, age displayed a positive correlation with left IMT and right IMT. This indicates that as age increases, the values of left IMT and right IMT increase.

The article "Correlation Analysis Between Required Surgical Indexes and Complications in Patients With Coronary Heart Disease" was retracted in 2023. Reasons: compromised peer review; false authorship; unreliable results or conclusions; concerns about the data.

**Table 2:** Pearson correlation analysis of age and IMT of the left common carotid artery and IMT of the right common carotid artery.

	Age	
Left common carotid artery IMT	Correlation coefficient	0.235*
	*p-value*	0.014
Right common carotid artery IMT	Correlation coefficient	0.238*
	*p-value*	0.012

*p < 0.05.

As shown in Table 3, analysis of variance (one-way analysis of variance) was used to study the differences between the types of CHD and the obtuse marginal branch of the left circumflex branch × 1, the middle segment of the right coronary artery (RCA) × 1, and the middle part of the left anterior descending branch × 1.5. Samples of different CHD types showed significance in the obtuse marginal branch of the left circumflex branch × 1, the middle part of the RCA × 1, and the middle part of the left anterior descending branch × 1.5. For non-ST-segment elevation angina pectoris with acute total vascular occlusion, the left circumflex artery is the most common, followed by the RCA and anterior descending branch.

**Table 3:** Analysis of variance between coronary heart disease type and obtuse marginal branch of the left circumflex branch, middle segment of right crown × 1, and middle part of the left anterior descending branch × 1.5 and total contrast scores.

	Type of coronary heart disease (mean and standard deviation)					*F*	*p*
	ST-segment elevation angina pectoris (*N* = 1)	Unstable angina pectoris (*n* = 124)	Stable angina pectoris (*n* = 9)	Ischemic cardiomyopathy (*n* = 56)	Non-ST-segment elevation angina (*n* = 25)		
Obtuse marginal branch of the left circumflex branch × 1	5.00 ± null	1.65 ± 1.19	1.71 ± 1.25	1.61 ± 1.17	2.17 ± 1.59	2.686	0.033*
Middle segment of the right coronary artery × 1	1.00 ± null	2.09 ± 1.37	1.29 ± 0.49	2.35 ± 1.49	2.91 ± 1.44	2.753	0.030*
Middle part of the left anterior descending branch × 1.5	1.00 ± null	2.50 ± 1.37	2.14 ± 0.69	2.59 ± 1.62	3.52 ± 1.27	3.084	0.017*

*p < 0.05; **p < 0.01.

As shown in Table 4, a variance analysis (one-way analysis of variance) was used to study the differences between the cardiac functional grade and the right IMT and the left IMT. As shown in Table 4, ultrasound of the carotid IMT in patients with CHD can predict changes in left ventricular function, but no specific correlation between left and right common carotid intima-media thicknesses was found.

**Table 4:** Variance analysis between the cardiac functional grade and the right intima-media thickness and the left intima-media thickness.

	Cardiac function classification (mean and standard deviation)				*F*	*p*
	Class I (*n* = 54)	Class II (*n* = 99)	Class III (*n* = 47)	Class IV (*n* = 15)		
Right intima-media thickness	0.87 ± 0.15	0.97 ± 0.22	0.94 ± 0.20	1.32 ± 0.37	8.174	*p *≤ 0.001**
Left intima-media thickness	0.88 ± 0.23	0.97 ± 0.22	0.98 ± 0.22	1.23 ± 0.14	4.694	0.004**

**p < 0.01.

The article "Correlation Analysis Between Required Surgical Indexes and Complications in Patients With Coronary Heart Disease" was retracted in 2023. Reasons: compromised peer review; false authorship; unreliable results or conclusions; concerns about the data.

As shown in Table 5, a variance analysis (one-way analysis of variance) was used to study the differences in the branch number of coronary vessel lesions with or without the presence of atherosclerotic cardiovascular disease (ASCVD). As shown in Table 5, samples with or without a medical history of ASCVD showed significance in the branch number of coronary vessel lesions. The value of the branch number of coronary vessel lesions in patients with ASCVD is higher than in those without ASCVD.

**Table 5:** Variance analysis of the branch number of coronary vessel lesions and medical history of atherosclerotic cardiovascular disease.

	Medical history of atherosclerotic cardiovascular disease (mean and standard deviation)		*F*	*p*
	No (*n* = 18)	Yes (*n* = 197)		
branch number of coronary vessel lesions	2.31 ± 1.03	2.80 ± 0.86	3.920	0.049*

*p < 0.05; **p < 0.01.

As shown in Table 6, a variance analysis (one-way analysis of variance) was used to study whether the presence of complications would affect the distal left circumflex branch × 1, the middle part of the left anterior descending branch × 1.5, and the distal left anterior descending branch × 1. As is shown in the table, whether there is any complication is significant with the distance of left circumflex branch × 1, the middle segment of left anterior descending branch × 1.5, and the distance of left anterior descending branch × 1. For patients without complications, the values of the distal left circumflex branch × 1, the middle left anterior descending branch × 1.5, and the distal left anterior descending branch × 1 were higher than those in patients with complications.

**Table 6:** Variance analysis for the presence of complications and distal left circumflex branch × 1, the middle part of the left anterior descending branch × 1.5, and the distal left anterior descending branch × 1.

	Complications (mean and standard deviation)		*F*	*p*
	No (*n* = 24)	Yes (*n* = 191)		
Total coronary angiography score	61.21 ± 48.26	38.31 ± 29.62	10.780	0.001**
Distal left circumflex branch × 1	2.74 ± 2.00	2.04 ± 1.45	4.243	0.041*
The middle part of the left anterior descending branch × 1.5	3.26 ± 1.42	2.54 ± 1.43	5.181	0.024*
Distal left anterior descending branch × 1	2.22 ± 1.91	1.60 ± 1.23	4.285	0.040*

* p < 0.05; **p < 0.01.

The article "Correlation Analysis Between Required Surgical Indexes and Complications in Patients With Coronary Heart Disease" was retracted in 2023. Reasons: compromised peer review; false authorship; unreliable results or conclusions; concerns about the data.

As shown in Table 7, correlation analysis was used to study the correlation between the VTE score and the proximal part of the RCA × 1, branch number of coronary vessel lesions, posterior descending branch of the left circumflex branch × 1, distal part of the left circumflex branch × 1, and middle part of the left anterior descending branch × 1.5, and the Pearson correlation coefficient was used to indicate the strength of the correlation. As shown in Table 7, the VTE scores showed a positive correlation with the proximal part of the RCA × 1, the branch number of coronary vessel lesions, the posterior descending branch of the left circumflex branch × 1, the distal part of the left circumflex branch × 1, and the middle part of the left anterior descending branch × 1.5. The higher the value of the VTE score, the higher the values of these six items.

**Table 7:** Pearson correlation coefficient of VTE scores and the proximal part of right coronary artery, the branch number of coronary vessel lesions, posterior descending branch of the left circumflex branch × 1, distal part of the left circumflex branch×1, and the middle part of the left anterior descending branch × 1.5

		VTE score
Proximal part of right coronary artery	Correlation coefficient	0.223**
	*p-value*	0.002
Branch number of coronary vessel lesions	Correlation coefficient	0.190**
	*p-value*	0.010
Posterior descending branch of the left circumflex branch × 1	Correlation coefficient	0.078
	*p-value*	0.294
Distal part of the left circumflex branch × 1	Correlation coefficient	0.174*
	*p-value*	0.018
Middle part of the left anterior descending branch × 1.5	Correlation coefficient	0.205**
	*p-value*	0.005

*p < 0.05; **p < 0.01.

## Discussion

The samples of different genders showed significant differences in the blunt marginal branch of left-handed branch × 1, diagonal branch of D1 × 1, and the manifestation of ms PV. Patients with left circumflex branch occlusion are mostly male and tend to be younger. In this sample, different genders showed significant differences in the blunt limb of the left branch × 1, the diagonal limb of D1 × 1, and the manifestation of ms PV. This statistically significant effect has been shown in other studies to be a statistically significant atherogenic effect on men (21); the risk status of men with coronary artery disease is more serious than that of women (22).

Age was positively correlated with the left IMT and right IMT, respectively. This indicates that with an increase of age, the left IMT and the right IMT increase. Due to the increase of minimum microvascular resistance, aging is related to the progressive panmyocardial injury of coronary vasodilation ability (23).

The article "Correlation Analysis Between Required Surgical Indexes and Complications in Patients With Coronary Heart Disease" was retracted in 2023. Reasons: compromised peer review; false authorship; unreliable results or conclusions; concerns about the data.

## Conclusions

A total of 215 patients (128 males and 87 females) with CHD were analyzed with SPSS. The obtuse marginal branch of the left circumflex branch, the diagonal branch, and the ms PV representative were analyzed by an independent-sample *t*-test in different ages and sexes. Complications of CHD and family medical history were analyzed through variance analysis, a chi-square test, etc. The study aimed to find the correlation between these variables.

In this sample,

(1) Samples of different genders showed significance in the obtuse marginal branch of the left circumflex branch × 1, the diagonal branch D1 × 1, and the ms PV representation. Patients with left circumflex branch occlusion are more male and tend to be younger.
(2) Age displayed a positive correlation with the left IMT and right IMT. This indicates that as age increases, the values of left IMT and right IMT increase.
(3) Samples of different CHD types showed significance in the obtuse marginal branch of the left circumflex branch × 1, the middle part of the RCA × 1, and the middle part of the left anterior descending branch × 1.5. For non-ST-segment elevation angina pectoris with acute total vascular occlusion, the left circumflex artery is the most common, followed by the RCA and anterior descending branch.
(4) Ultrasound of the carotid IMT in patients with CHD can predict changes in the left ventricular function, but no specific correlation between left and right common carotid intima-media thicknesses was found.
(5) Samples with or without a medical history of ASCVD showed significance in the branch number of coronary vessel lesions. The value of the branch number of coronary vessel lesions in patients with ASCVD is higher than in those without ASCVD.
(6) Whether there is any complication is significant with the distance of left circumflex branch × 1, the middle segment of left anterior descending branch × 1.5, and the distance of left anterior descending branch × 1. For patients without complications, the values in the distal left circumflex branch × 1, the middle left anterior descending branch × 1.5, and the distal left anterior descending branch × 1 were higher than those in patients with complications.
(7) The VTE scores showed a positive correlation with the proximal part of the RCA  × 1, the branch number of coronary vessel lesions, the posterior descending branch of the left circumflex branch × 1, the distal part of the left circumflex branch × 1, and the middle part of the left anterior descending branch × 1.5. The higher the value of the VTE score, the higher the values of these six items.

The article "Correlation Analysis Between Required Surgical Indexes and Complications in Patients With Coronary Heart Disease" was retracted in 2023. Reasons: compromised peer review; false authorship; unreliable results or conclusions; concerns about the data.

## Data Availability

The original contributions presented in the study are included in the article/supplementary material, further inquiries can be directed to the corresponding author/s.
